# The Impact of Wireless Network Mobile Devices on College Students' Labour Concept Education in Artificial Intelligence Environment

**DOI:** 10.1155/2022/4714445

**Published:** 2022-03-26

**Authors:** Jingmin Li

**Affiliations:** Experimental Training Management Center, School of Jilin Business and Technology College, Changchun, China

## Abstract

To cultivate correct labour values and good labour quality of college students and effectively promote the development of their labour concept education, this work explores the impact of wireless network mobile devices on college students' labour concept education under the environment of artificial intelligence. Firstly, a questionnaire survey is used to investigate the labour concept of 400 college students. Secondly, the impact of wireless network mobile devices on college students' labour education is obtained by comparing group A (using artificial intelligence APPs for wireless network devices to learn about labour concepts) and group B (using traditional classroom teaching methods for to learn about labour concepts). According to the statistical survey results, about 20% of college students agree that “if they have enough money to live, they do not have to work”; while less than 50% agree that “they cannot be admitted to civil servants and senior managers in the company and are willing to engage in ordinary labour in the future”. Meanwhile, about 50%–60% of college students think that “housework has nothing to do with me, and it's all the work of adults”. In the question “What would you do when you find that the public area is dirty and poor, but it's not your turn to be on duty?”, only about 50% of college students are willing to clean actively. Comparing the data of group A and group B suggests that the labour view expressed in group A is more biased in the cognition of labour purpose, and students in group A is more negative and lazier in labour attitude and labour habits, which shows that wireless network mobile devices have a great negative impact on the overall labour view of college students. Therefore, it is revealed in this work that the correct use of artificial intelligence technology in the education of labour concept has extremely important value for the intelligent development of education methods.

## 1. Introduction

With the rapid development and wide application of artificial intelligence, it has had a profound impact on human labour and brought earth-shaking changes to human society. Artificial intelligence not only affects the human labour concept and changes human labour mode, but also widens the scope of human labour and enriches the content of human labour. The continuous development of artificial intelligence not only replaces part of human labour but also reduces the opportunities for college students to work, resulting in limitations in college students' cognition of labour concept education [1]. Contemporary college students' labour consciousness is generally weak. They yearn for a comfortable life, are content with the current situation, and lack a correct understanding of the concept of labour [2]. It is caused by many factors. Among the various factors, network mobile devices that have been gradually popularized among college students, such as mobile phones and computers, play an important role in transmitting information through network media. They are influenced by social network hot news, such as stars' sky-high film pay, online popularity, fame, and wealth. Many college students believe that they can get a high income without hard work, which has an impact on college students' world outlook, attitude about life, and values. In addition, college students' conception of labour has also deviated [3, 4].

At present, foreign research on labour concept education mainly refers to the concept of labour education. Many scholars agree that labour education helps promote the all-around development of college students, and they believe that labour is the essence of mankind. Labour education has important value for promoting the all-around development of college students. Its value is mainly reflected in helping college students establish correct labour values, providing ideological guarantees for the all-around development of college students and giving full play to the comprehensive educational function. Besides, labour education promotes the harmonious physical and mental development of college students [5]. Many scholars have conducted research on the content of labour concept education. House et al. (2019) discussed how the Toronto Labour Council can provide a space for socialist-led workplace organisational training and political education; and finally, the possible role of the labour concept education of the committee model in the revival of the socialist movement was discussed [6]. Chen and Xie (2020) used labour concept, labour skills, and labour consciousness as independent variables and labour habits as dependent variables for analysis and established a regression model to predict the labour habits of college students. The results revealed that there is a significant correlation between labour awareness, labour concept, labour skills, and labour habits, and there is a strong positive correlation, which provides support for colleges and universities to cultivate college students' labour habits [7]. Chen (2020) analyzed the controversy, degree of deformation, and quantitative evaluation of labour education ideas and discussed how to link labour education with labour ideas and labour harvests to form a closed-loop structure, making labour education endless [8]. Gao et al. (2020) believed that promoting the integration of “labour major” education in colleges and universities, by strengthening education on labour values, building an evaluation index system for the “labour major” integrated education mechanism, and establishing a scientific and reasonable evaluation index system. In this way, measures such as effective integration and training of “integrated” teachers could be realized, and the value of “labour-vocation” integrated education was reflected in college education [9]. Although many scholars have conducted many studies on labour concept education, there is little research on the impact of wireless network mobile devices on college students' labour concept education in the artificial intelligence environment. Exploring and analysing the specific impact of wireless network mobile devices in college students' labour concept education is of great significance for seeking positive and effective correction methods.

The objective of this work is to create a good working atmosphere among college students, promote college students to form a consciousness of respecting and loving labour, and establish a correct view of labour. The innovation of this work is that it tries to analyze the impact of artificial intelligence APPs in wireless network mobile devices on the education of college students' concept of labour by means of questionnaires. The questionnaire investigates the cognition of labour purpose, labour meaning, labour division, labour awareness, labour attitude, and labour habits of college students. Finally, the correct use of artificial intelligence technology in labour concept education will provide a path to explore based on the survey results.

## 2. Materials and Methods

### 2.1. Analysis of the Current Situation and Influence of Labour Concept Education under the Background of Artificial Intelligence

In the process of labour, people will always form their views and understanding of labour, which is the concept of labour. The concept of labour reflects the attitude of workers towards labour and determines the behaviour of workers in the process of labour [10]. Whether the concept of labour is correct or not is directly related to whether people can establish a correct outlook on life, world outlook, and values. Only by establishing a correct outlook on work can a person consciously strengthen the awareness of the most glorious of hard work, create life with both hands and wisdom, realize his ideals, and play a positive role in the formation of outlook on life and world outlook [11, 12].

The education of labour concept is to train the educated to establish correct labour concept and labour attitude, develop the emotion of loving labour and working people, cultivate good labour habits, and have innovative and creative labour quality [13, 14]. The labour concept education of college student is to cultivate college students to establish a scientific labour cognition, correct labour attitude, establish a correct labour value orientation, respect the working people, cherish labour achievements, and form a good habit of loving and innovating labour [15]. The labour outlook education of college students is an important part of ideological and political education, which plays a very important role in establishing a correct outlook on life, world outlook, and values for college students [16].

The concepts of labour education and labour concept education are different, but they are related to each other. Labour education includes labour concept education, which is an important part of labour education [17, 18]. The connotation of labour education is relatively broad, including both labour technology education and labour moral education [19]. From the perspective of ideological and political education, labour concept education is the core content of labour education. Although labour knowledge education and labour skill education belong to the content of labour education, they do not belong to the content of labour concept education. However, labour knowledge education and labour skill education are important means to promote labour concept education. Positive labour knowledge education and labour skill education help to promote the realization of labour concept education [20].

Under the background of artificial intelligence, the connotation of college students' labour concept education mainly includes labour attitude education, labour spirit cultivation, labour values education, and labour habit cultivation. Labour attitude mentions three aspects: labour cognition, labour emotion, and labour intention. Labour attitude is oriented, determines what kind of psychology people adopt to implement labour behaviour, and plays a directional guiding role in people's labour behaviour [13].

The working spirit is the positive expression of the working people in the concept and practice of labour. It shows the spirit of workers' love for labour and hard work and reflects the value orientation of a nation. Labour values refer to people's judgment of labour value and the view that labour creates value. Labour habit refers to an instinctive way of behaviour gradually formed in the process of long-term labour. It is an independent and conscious action. The cultivation of labour habits plays a vital role in the cultivation of college students' labour ability.

### 2.2. Experimental Object and Experimental Process

This work adopts the way of questionnaire to explore the impact of wireless network mobile devices on college students' labour concept education under the environment of artificial intelligence. The questionnaire sample selects 400 college students from a university and divides them into group A and group B. Among them, 200 college students in group A used the artificial intelligence APPs of wireless network equipment to study the content related to the concept of labour; while 200 college students in group B used traditional classroom teaching methods to study the content related to the concept of labour. The questionnaire investigates the concept of labour education from college students' cognition of labour purpose, labour significance, division of labour, labour consciousness, labour attitude, and labour habits.  Figure 1 shows the flow chart of a questionnaire survey experiment.

### 2.3. Reliability Test of the Questionnaire

Reliability refers to the consistency, stability, and credibility of test results. The higher the reliability coefficient is, the more consistent, stable and reliable the test results are. Reliability refers to the consistency of the results when the same method is used to measure the same object repeatedly. On the other hand, reliability refers to the credibility of measured data [21, 22]. The commonly used reliability measurement index is the Cronbach α coefficient [23], which is calculated as follows:

(1) $$\begin{array}{c} \alpha =\frac{K}{K-1}\left(1-\frac{\sum_{i=1}^{K}\sigma_{\gamma^{i}}^{2}}{\sigma_{X}^{2}}\right). \end{array}$$

In (1), *K* is the number of questions in the questionnaire; *σ*_*X*_^2^ is the variance of the total test score; and *σ*_*γ*^*i*^_^2^ is the score variance of question *i*.

According to the definition of the Cronbach coefficient *α*, its calculation equation can also be expressed in the form of variance.

(2) $$\begin{array}{c} \alpha =\frac{\sigma^{2}\left(p\right)}{\sigma^{2}\left(p\right)+\sigma^{2}\left(pi\right)/n}. \end{array}$$

In (2), *σ*^2^(*p*) is the estimated value of the true fractional variance component, *σ*^2^(*pi*) is the variance component of relative decision error, and *n* is the number of items.

(3) $$\begin{array}{c} \alpha =\frac{MS\left(p\right)-MS\left(pi\right)}{MS\left(p\right)}. \end{array}$$

In (3), MS(p) is the true fractional mean square and MS(pi) is the error mean square.

In this work, SPSS 26.0 is used to analyze the data obtained from the questionnaire. *α* is between 0 and 1. The reliability corresponding to different values is shown in Table 1 [24, 25].

## 3. Results and Discussion

400 questionnaires were distributed in this experiment. 198 questionnaires were recovered in group A, with a questionnaire recovery rate of 99%, and 195 papers were recovered in group B, with a questionnaire recovery rate of 97.5%. The analysis of the reliability of the questionnaire shows that the Krabaha coefficient of this questionnaire is 0.869. This indicates that the questionnaire designed shows strong internal consistency and stability and high reliability, indicating that the reliability of the questionnaire design can be used for research analysis.

### 3.1. Impact of Wireless Network Mobile Devices on College Students' Cognition of Labour Significance and Labour Purpose

An important aspect of labour concept education for college students is to let them know the significance of labour. The questionnaire on the meaning of labour mentions the following five answers. (1) Labour is the precondition for human survival and development. (2) Labour creates human and human society. (3) Labour can achieve human liberation and promote the comprehensive and free development of human beings. (4) Labour is a measure of the value of life. (5) Happiness is achieved through struggle.  Figure 2 shows the statistics of the percentage of college students who agree with these views, and the corresponding meanings of the numbers on the abscissas.

Figure 2 shows that about 75% (74.67% in group A and 75.58% in group B) of students agree that labour is the prerequisite for human survival and development and about 65% (67.25% in group A and 65.77% in group B) agree that labour creates people and human society. Besides, about 60%–64% (61.91% in group A and 64.28% in group B) of college students agree that labour can realize people's liberation and promote people's all-around and free development. Meanwhile, about 60%–63% (60.51% in group A and 63.19% in group B) of college students agree that labour is the measure of life value. In addition, about 73%–76% (63.64% in group A and 67.54% in group B) of college students struggle for happiness. Comparison on the survey results of group A and group B suggests that the cognition of the two groups of college students on the purpose of labour is basically the same, indicating that wireless network mobile devices have little impact on college students' labour significance.

For the investigation of college students' cognition of labour purpose, the two viewpoints of “labour is to earn more money” and “if you have enough money to live, you do not have to work” are selected to understand the cognition. Figures 3 and 4 illustrate the survey results. The abscissa “1” in the figure indicates “identity” and “2” indicates “comparative identity,” “3” means “neutral,” “4” means “not quite disagree,” and “5” means “disagree”.

It can be observed from Figure 3 that if college students agree with the questions set in the questionnaire as measured by “identity” and “comparative identity”, and disagree with “not quite identity” and “not identity”, more than 60% of college students agree with “labour is to earn more money”, and less than 10% of college students disagree. It shows that college students have a high recognition of “labour is to earn more money”. Comparing the survey results of group A and group B, it is found that the cognition of the two groups of college students is basically the same, but Figure 4 illustrates that only about 20% of them agree that “if they have enough money to live, they do not have to work”. Comparing group A and group B reveal that group A has a higher degree of approval for this view, reaching 26.98%, indicating that the use of wireless network mobile devices has a negative impact on college students' view of labour. On the whole, there is a certain degree of deviation in college students' cognition of labour purpose, and the use of wireless network mobile devices aggravates this cognitive deviation.

### 3.2. Impact of Wireless Network Mobile Devices on College Students' Division of Labour and Labour Awareness

Division of labour refers to the division, independence, and specialization of people's socio-economic activities. Its purpose is to make workers engaged in all walks of life more professional, so as to improve labour productivity and create more wealth [26]. For the investigation of college students' cognition of division of labour, two viewpoints were selected to understand the cognition: “the labour of farmers and workers is as respectable as that of scientists” and “if they cannot be admitted to civil servants or senior managers of the company, they are willing to engage in ordinary labour work in the future”. Figures 5 and 6 reveal the survey results. The abscissa “1” in the figure means “agree,” “2” means “relatively agree,” “3” means “neutral,” “4” means “not quite agree,” and “5” means “disagree”.

According to the survey results in Figures 5 and 6, if college students agree with the questions set in the questionnaire as measured by “agree” and “relatively agree,” and disagree with “not quite agree” and “disagree”. About 70% (67.61% in group A and 72.46% in group B) of college students agree when asked about “the labour of farmers and workers is as respectable as that of scientists”. The recognition of the other question “if you cannot be a civil servant or a senior manager of the company, you are willing to engage in ordinary labour work in the future” is less than 50% (48.61% in group A and 53.43% in group B). Compared with group A and group B, it is found that group A has relatively low recognition of the view that “if you cannot be a civil servant or a senior manager of the company in the future, you are willing to engage in ordinary labour work”. It shows that unlimited network mobile devices have a negative impact on college students' cognition of division of labour.

For the investigation of college students' cognition of labour consciousness, the view of “if you want to obtain wealth, you must work” is selected to understand cognition. The survey results are shown in Figure 7. The abscissa “1” in the figure indicates means “agree”, “2” means “relatively agree,” “3” means “neutral,” “4” means “not quite agree,” and “5” means “disagree”.

It is found in Figure 7 that both group A and group B have more than 80% (88.10% in group A and 83.33% in group B) recognition of the view that “if you want to obtain wealth, you must work” (both “agree” and “relatively agree” mean recognition), and less than 10% (4.13% in group A and 5.87% in group B) disapproval (both “not quite agree” and “disagree” mean disapproval), which shows that contemporary college students have a strong sense of labour. Compared with group B, students in group A show slightly higher recognition on this issue, which may be due to the positive impact of some smart apps used in wireless network mobile devices, such as learning power. It has a positive impact on strengthening college students' labour consciousness.

### 3.3. Impact of Wireless Network Mobile Devices on College Students' Cognition of Labour Attitude and Labour Habits

Labour attitude refers to people's stable psychological tendency towards labour formed on the basis of ideas. The survey on college students' cognition of labour attitude chooses “housework has nothing to do with me, and it's all adults' work”. This view is used to understand the cognitive situation.  Figure 8 suggests the survey results. When analysing the survey results, both “agree” and “relatively agree” indicate approval, and both “not quite agree” and “disagree” indicate disapproval.

Figure 8 illustrates that nearly 50%–60% (59.67% in group A and 53.93% in group B) of college students in group A and group B think that “housework has nothing to do with me, and it's all the work of adults”. It further shows that only about 15%–20% (17.11% in group A and 23.23% in group B) of college students do not agree with this view. Obviously, the recognition of this issue is somewhat high, which shows that most college students have a lazy attitude towards labour. Comparing group A and group B, group A has a higher recognition of this problem. It may be caused by the use of unlimited network mobile devices, which leads to the negative labour attitude of college students. Under the negative influence, students usually escape from labour and have high standards but do not pay for practice.

Labour habit refers to an instinctive way of behaviour gradually formed by people in the process of long-term labour [27]. For the survey of college students' cognition of working habits, the question is “What would you do when you find that the public area is dirty and poor, but it's not your turn to be on duty?” Figure 9 shows the survey results. In the abscissa, “1” means “active cleaning”, “2” means “remind the students on duty to clean”, and “3” means “indifference”.

According to the cognitive survey results of college students' working habits in Figure 9, when asked “What would you do when you find that the public area is dirty and poor, but it's not your turn to be on duty?” When this question is asked, more than 50% of the students will choose to take the initiative to clean, more than 30% of the students choose to remind the students on duty to clean, and the remaining students choose to be completely indifferent. Compared with group A and group B, it is found that fewer college students in group A choose to take the initiative to clean and have poor working habits.

### 3.4. Discussion

The comparative analysis of the results obtained in group A and group B reveals that, on the whole, some smart APPs in the use of wireless network mobile devices, such as learning to strengthen the country, have had a positive impact on strengthening the labour awareness of college students. Therefore, in the follow-up colleges and universities to carry out labour concept education, they should face the impact of artificial intelligence technology rationally.

First of all, the curriculum content of labour concept education can be enriched by strengthening curriculum construction. On the one hand, universities and colleges should organically integrate labour concept education into ideological and political courses. On the other hand, education on the concept of labour also needs to add elements of the times and incorporate relevant knowledge of artificial intelligence. Combining the knowledge of artificial intelligence with the content of labour concept education makes labour close to real life, which is conducive to breaking the image of labour in the minds of college students [28]. The educational content of the concept of labour should be updated in time with the changes of the times, not only to convey the labour theory to college students, but also to popularize the relevant background knowledge of artificial intelligence to realize a new round of knowledge transformation [29]. Therefore, the curriculum content of labour concept education of college students should closely follow the theme of the times, and practically achieve “everything from reality” to better meet the labour needs of the era of artificial intelligence.

Second, innovate classroom teaching methods can use artificial intelligent methods to impart theoretical knowledge. On the one hand, teachers can use intelligent technology and intelligent software in the course of teaching to carry out modern, intelligent and personalized teaching for college students, and highlight knowledge points in a targeted manner. On the other hand, on the basis of the traditional teaching methods in the classroom, the classroom teaching methods are innovated for heuristic teaching, discussion teaching, interactive teaching, and dialogue teaching for college students. For example, the intelligent system is used to match individualized learning methods and learning content for each college student, so that the teaching quality and efficiency of teachers can be effectively improved.

Finally, the artificial intelligence technology is adopted to set up labour practice teaching and create an intelligent social practice platform. Using artificial intelligence technology can help schools set up labour practice teaching, so that labour practice learning becomes a part of daily life of college students. Participating in labour practice is a transition from brain to hands-on, from in-class to out-of-class, from theory to practice, and ultimately improves the thinking and ability of creative labour during labour time [30, 31].

## 4. Conclusion

With the continuous development of artificial intelligence, wireless network mobile devices are gradually popularized among college students. The information transmitted through network media imperceptibly affects the labour view of contemporary college students. According to the statistical results of the questionnaire survey, most of the students hold the attitude of “working to earn more money”, but show indifference to housework, which indicates that there are some problems in the view of labour of contemporary college students that cannot be ignored. The concept of labour expressed is relatively biased in the cognition of the purpose of labour, and there are obvious differences in knowledge and action in the division of labour, which suggests that the application of artificial intelligence technology in the education of labour concept should be further changed, so that it can have a positive impact on the overall understanding of college students on labour. There are many reasons for the above views in the education of labour concept of college students. However, in this work, there are also some shortcomings, such as the sample size of this questionnaire is not sufficient due to time constraints. Therefore, in the future work, the sample size will be further increased to make the obtained results more credible, and other influencing factors that affect the education of college students' outlook on labour will be explored.

## Figures and Tables

**Figure 1:** Flow chart of a questionnaire survey experiment.

**Figure 2:** Survey results of college students' cognition of labour significance.

**Figure 3:** Survey results of college students' cognition of labour purpose (“labour is to earn more money”).

**Figure 4:** Survey results of college students' cognition of labour purpose (“if you have enough money to live, you do not have to work”).

**Figure 5:** Survey results of college students' cognition of division of labour (“The labour of farmers and workers is as respectable as that of scientists”).

**Figure 6:** Survey results of college students' cognition of division of labour (“if they cannot be admitted to civil servants and senior managers of the company in the future, they are also willing to engage in ordinary labour work”).

**Figure 7:** Survey results of college students' cognition of labour consciousness.

**Figure 8:** Survey results of college students' cognition of labour attitude.

**Figure 9:** Survey results of college students' cognition of working habits.

**Table 1:** Reliability degree corresponding to *α* values.

Krabaha coefficient (*α*)	Reliability
0.9 <*α*< 1	Higher
0.8 <*α*< 0.9	Suitable for research and analysis
0.7 <*α*< 0.8	Lower

## Data Availability

All data are available from the corresponding author upon request.
